The article "Skeletal Structure and Training Adaptability of Athletes Based on Biomechanical Analysis" was published in 2022. Journal: J Healthc Eng.

# Skeletal Structure and Training Adaptability of Athletes Based on Biomechanical Analysis

**DOI:** 10.1155/2022/3083821

**Published:** 2022-02-15

**Authors:** Xiaoqin Yin, Lili Wang, Lan Zhang

**Affiliations:** Department of Physical Education, Shihezi University, Shihezi 832003, Xinjiang, China

## Abstract

According to the kinematics analysis of the human body, a set of exoskeleton mechanical structures is designed to imitate the physiological structure and movement characteristics of the lower limbs of humans. To study the biomechanical characteristics of the exoskeleton in two different phases during walking and to provide a research basis for the design and optimization of the exoskeleton. Doctors and engineers are actively committed to the basic understanding and improvement of the tissue characteristics, structure, and function of the human musculoskeletal system. Firstly, according to the gait analysis of the lower limbs, the exoskeleton mechanical structure is designed by using three-dimensional modeling software. After the solid model is generated, the assembly, meshing, and element attribute assignment are carried out by using finite element software. And the face-to-face contact relationship between each building is established, and the stress distribution of the exoskeleton is simulated and analyzed. The stress distribution of the exoskeleton under different working conditions is significantly different. Since the calculation does not take into account uncertainties such as shocks that may occur during walking, it is necessary to consider and multiply a certain safety factor when designing the optimized exoskeleton.

## 1. Introduction

The human body's motion system consists of three major organs: muscle, bone, and joint. It is the central content of the force, lever, and fulcrum in the human body's motion system [1]. The combination of structure and function of the three originated from the embryo. After birth, bones are continuously modeled and remodeled due to their adaptation to the external environment, especially to mechanical stimuli [2]. Sports injuries are a basic problem that plagues athletes. Understanding the mechanism of sports injury and its prevention is not only a basic problem of sports medicine, but also one of the basic problems of our research on sports biomechanics [3]. At present, most of the domestic research on exoskeletons is based on the control field, and there are few studies on the external bone mechanical structure, and the rationality of the exoskeleton mechanical structure design directly determines the performance of the whole system. In recent years, with the continuous advancement of digital and computer technology, the finite element method has become an extremely useful tool for analyzing changes in orthopedic mechanics. The simulation conditions are closer to reality, and the reliability of the results is higher [4]. Exercise, as an effective means to enhance bone quality, has been widely used. The influence of exercise on bone biomechanical properties has become one of the hotspots in sports medicine. On the basis of consulting relevant literature, this paper reviews the effects of different exercise modes on bone biomechanical properties and its research progress. In order to improve the biomechanical properties of bone, choose a better way of exercise and strength to improve the scientific basis and reference [5]. Since 2014, the research theory of an optimized core shell polymer nanofiber membrane in the gel polymer electrolyte has been put forward [6]. After that, the theory of the preparation of oil in water emulsion by three-dimensional double continuous skeleton hydrophobic polymer film was also proposed by [7]. In 2016, the theory of the effect of temperature on the mechanical properties of mullite fiber ceramics with a three-dimensional framework fabricated by moulding was studied by relevant scholars [8].

In the process of bone tissue metabolism, bone formation and bone remodeling are continuously carried out under the stimulation of the outside world. Exercise can improve the quality of bone, enhance the ability of bone to resist fracture, and reduce the risk of fracture [9]. Chinese scholars have elaborated on the research of the finite element method of biomechanics in some disciplines from their respective specialties, but they lack systematization. In this paper, the concept and principle of the finite element method and the scope and progress of finite element research in skeletal biomechanics are reviewed [10]. The exoskeleton is a new mechanical booster similar to an insect exoskeleton, which aims to help people expand their lower limb movement ability. It can help individual soldiers to increase their abilities to bear heavy loads, enhance the sports ability of disaster relief and explosion-proof personnel, and help the elderly and disabled people to improve their ability to live independently. [11]. In addition to the influence of heredity, age, and gender, bone mass is also regulated by mechanical load, hormones, and nutrition. The human body needs to do basic exercise to maintain bone mass, and the use of or no weight causes a significant decrease in bone mass [12]. The basic idea is to simulate the human skeleton frame and transfer the load to the ground through the exoskeleton to reduce the load on the human body. From the perspective of biomechanics, this paper focuses on the structural and functional adaptation of skeletal muscle to explore the mechanism of skeletal muscle motor injury, aiming to inspire the jade and work on deep human research in this aspect of sports biomechanics [13].

Bone biomechanics is considered to be one of the most leading branches of biomechanics, and it has made countless epoch-making contributions to the biological sciences, medicine, industry, and even our daily lives. The biomechanical properties of bone include structural mechanical properties and mechanical properties of materials [14]. The structural mechanical properties of bone refer to the mechanical properties of the entire bone structure, which are related not only to the mechanical properties of the bone but also to the geometrical properties of the bone. That is, the influence of shape, size, etc. on the structural mechanical properties of the bone can be reflected by the load-deformation curve. The human body weight exoskeleton is a human-computer integrated system. In the process of walking, wearability and comfort are the primary considerations [15]. In order to design a comfortable exoskeleton, it must be based on an important principle—anthropomorphic. Chinese scholars have elaborated on the research of the finite element method of biomechanics in some disciplines from their respective specialties, but there is a lack of systematization [16]. In this paper, the concept and principle of finite element method and the scope and progress of finite element research in skeletal biomechanics are reviewed. The material mechanical properties of bone refer to the mechanical properties of bone tissue itself, which are independent of the geometric shape of bone. The material mechanical properties of bone can be reflected by stress-strain curves [17]. This paper mainly outlines the mechanism of adaptive change and regulation of mechanical stimulation (stress) or physical exercise on bone-bone mineral density and structure and briefly introduces the modern measurement techniques and methods of related research and evaluation indicators [18].

This paper summarizes the adaptability of bones to the external environment and especially introduces the adaptive changes and related mechanisms of bones to mechanical stimuli related to exercise, as well as the measurement and evaluation techniques and methods of modern bone research. The innovative contributions of this paper include the following: 1. The repair effect of muscle strain is limited by the degree of muscle injury and the treatment of muscle injury. 2. In the exoskeleton design, the principles of human kinematics are analyzed and the joint design of human bone connection is simulated. 3. When the mechanical load applied to the bone increases, the strain of the bone increases. When the strain increases to or exceeds a certain limit, it stimulates the bone to start the bone reconstruction process.

## 2. Materials and Methods

Each muscle is wrapped by a dense deep fascia, such as the “tightly fitting” structure. The deep layer of the deep fascia is the denser epimyocardium. The muscles are divided into several parts called muscle bundles, and the membrane structure surrounding the muscle bundles is the muscle peritoneum [19]. The sequence of human lower limb walking is the division of dynamic walking in time series, and it is the basic theory to study walking characteristics [20]. Only by clearly analyzing the movement laws of human lower limbs can we further design the joint freedom of lower limbs. The walking of the human body is the circular motion of its lower limbs, and a complete cycle becomes a step. A step consists of a supporting phase and a wobble phase [21]. The material toughness of bone refers to the area under the stress-strain curve, which indicates the energy required to cause fracture of the bone material and is affected by changes in bone matrix composition such as bone mineral content and collagen fiber orientation. Bone tissue with higher toughness can better resist the occurrence of fractures, and the toughness of bone decreases with age. The acquired factors have a great influence on the growth and development of the bone, the peak bone mass, and the process and severity of osteoporosis. The effect on the peak bone mass is particularly significant. After reaching the peak bone mass (about 30 years old), the bone mineral density of men and women decreases with age, and the elastic modulus and strength of dense bone also decrease, and women are more prominent than men.

Table 1 lists the range of activities of the exoskeleton. In general, this range of activities is greater than the range of activities of a person while walking and less than the maximum range of activities of a person.

In case 1, the exoskeleton is symmetrical, so the stress of the left and right legs is the same. Only half of the results need to be extracted when extracting the results. The stress calculation results of each component are shown in Table 2.

Start the PID_ILC control program written in MATLAB, generate the new motor 3, 4 input displacement curves, save Excel as the input of the next operation, and repeat the process. The initial states of A and B are shown in Figures 1 and 2.

The main interstitial component of muscle health is collagen fibers. Collagen fibers interweave into bundles, which are surrounded by a layer of loose connective tissue touching the intima, slipping slightly between the bundles of collagen fibers, with blood vessels and lymphatic vessels running among them [22]. Outside the muscle cavity, there is also a complete adventitia, which is connected with the endometrium. From the point of view of mechanism, the lower limb skeletal kinematic chain is a series-parallel hybrid structure with rotational motion as its main component. According to the different forms of lower limb movement, it shows different forms of movement chain. Considering the activities of each joint, the motion of the human lower limbs is positioned at 7 degrees of freedom. The effect of exercise on bone mechanical properties increases with the increase of exercise intensity. The effect of moderate load exercise on bone mechanical properties is greater than that of low load exercise. Therefore, it was concluded that in order to obtain an increase in bone mass, a large exercise load suitable for the individual should be selected under the critical strength load. The alteration of the dense bone with age will result in a compensatory increase in the transverse moment of inertia of the backbone, thereby reducing the decrease in bone strength due to the reduction in bone density. This also explains why senile osteoporotic fractures often occur in the spine, the proximal femur, and the distal radius of the humerus. Periorbital tissue formed by loose connective tissue reduces friction between the muscle bond and its surrounding tissue. When viewed with a polarizing microscope, the muscles exhibit a curled, wavy appearance. The way in which the muscle bond is crimped plays an important role in its mechanical properties, and degenerative aging changes are seen very early in the tendon tissue.

## 3. Result Analysis and Discussion

To design the external bone mechanical structure, we must first understand the force transmission mechanism and mechanics of the exoskeleton, including the force characteristics of the exoskeleton in the unsynchronized state. After analyzing the human gait, the legs were selected, the left toe was off the ground, and the vertical critical point of the tibia was taken as the calculation condition. Since the two feet stand and the left toe are similar to the ground, so the standing position of the legs and the vertical critical point of the tibia are finally taken as the calculation conditions. In the metabolic process of bone tissue, exercise as a mechanical load has an effect on the biomechanical properties of bone, but too low a load is insufficient to cause adaptive changes in bone. The effect of excessively high loads and easy-to-cause bone resorption is greater than the effect of bone formation, resulting in a negative balance of bone metabolism. As a result, bone loss and bone biomechanical properties are reduced, so that proper exercise can better improve and improve bone mechanical properties. The exogenous mechanical forces exerted on the skeleton after birth can be summarized as endogenous muscle contraction force and exogenous reaction force, even if the bone deforms. These forces regulate bone growth and development mainly by regulating intrachondral growth and ossification, articular cartilage development, perichondral/periosteal ossification, and intrachondral osteogenesis. In the process of muscle stretch and contraction, it undertakes the important functions of energy absorption, protection of muscle fibers, and force transmission and is the important structural basis for the functional realization of muscle organs. With the influence of training load, the structure and function of the membrane and key structure system will change adaptively. Therefore, the membrane system and cavity structure cannot be ignored in strength training.

In the simulation experiment, the initial state of iterative learning is shown in Figure 3. After nine iterations, the output curve of the model converges to the target curve (Figure 4). The convergence process of the whole iterative learning is shown in Figure 5.

In calculation condition 2, the left and right sides of the exoskeleton are no longer symmetrical, and the stress results of each component need to be extracted separately. The calculation results are shown in Table 3.

Binary coding is adopted in the coding mode, the roulette selection operator is used in the selection operator, the single point crossover operator is used in the crossover operator, and the basic bit mutation operator is used in the mutation operator. Other calculation parameters are shown in Table 4.

For the mass of the external load *f*, the acceleration of motion is *b*, which is known according to Newton's second law:

(1) $$\begin{array}{c} f^{\prime }=af+b. \end{array}$$

It can be seen that changes in muscle strength can be obtained by changing either mass or acceleration, using the following mathematical expressions:

(2) $$\begin{array}{c} f\left(x\right)=\frac{1}{g\left(x\right)},\\ f^{\prime }=f-\left(\bar{f}-c\sigma \right). \end{array}$$

The process of progressively contacting the foot with the ground is seen as a parallel loading of a spring-damped system:

(3) $$\begin{array}{c} f_{\max}^{\prime }=C_{\text{mult}}\cdot f_{\text{avg}}. \end{array}$$

Think of this process as the torque balance of the ankle around the ankle.

(4) $$\begin{array}{c} k_{i}=A_{i}\exp\left(-\frac{\Delta E_{i}}{RT}\right). \end{array}$$

The process 1 and 2 reaction forces are superimposed, and the relationship between the resultant forces *x* and *e* and the motor 3 displacement ax can be obtained by appropriate simplification:

(5) $$\begin{array}{c} F\left(x\right)=\frac{1}{1+e^{-ax}},\\ o_{j}\left(t\right)=f\left(\left[\sum_{i=1}^{n}w_{ij}x_{i}\left(t-\tau_{ij}\right)\right]-T_{ij}\right). \end{array}$$

The most common one in the iterative learning algorithm is the proportional integral derivative (PID) type. Its parameter concept is clear, and it can guarantee convergence and have a fast convergence speed through reasonable tuning. Its form is as follows:

(6) $$\begin{array}{c} Y_{j}\left(t\right)=\phi \left(\sum_{i=1}^{n}w_{ji}x_{i}-\theta_{j}\right). \end{array}$$

The effect of each iterative learning is evaluated by the root mean square (RMS) error, which reflects the degree to which the measured data deviates from the true value (including the positive and negative deviations) and is an indicator for evaluating the tracking of the trajectory.

(7) $$\begin{array}{c} P_{i}=\frac{f_{i}}{\sum_{i=1}^{N}f_{i}},\\ CI_{i}=\frac{\sum_{j}\left(C_{ij}/\left(C/N\right)\right)\ln\left(C_{ij}/\left(C/N\right)\right)}{N\;\ln\left(N\right)}. \end{array}$$

The vertical ground reaction force output A shown in Figure 6 is similar in shape to the M-shaped curve obtained in the actual system, indicating that the model basically reflects the laws of the actual system.

Muscle strength refers to the ability of muscle contraction to overcome internal and external resistance during human motor activity. Internal resistance includes the gravity of the human body, the reinforcing force of the joint, the viscous force of the muscle ligament, and the reaction force inside the human body (inertial force); external resistance includes gravity, supporting reaction force, friction force, medium resistance, inertial force, and the like. Considering that the three-dimensional finite element method has been widely used in mechanical properties research in recent years, in order to verify whether the design scheme meets the design requirements and finally determine the design result, ANSYS software is used for numerical simulation. The entire construction geometry model is more complicated, so Hypermesh is used for geometric processing and meshing. The two software structures are used to import the mesh into ANSYS, and the joints are analyzed by face-to-surface contact elements. At present, this process can also perform computer finite element stress analysis and simulation through a “continuous bone material model.” However, in order to verify the local or comprehensive effects of mechanics on bone mass, that is, to determine the “end-pint measure,” it is necessary to establish animal models or to compare and evaluate different exercise loads on human beings. It changes with the human body's functional state and a reasonable degree of exertion. External resistance is the exerting factor and means of strength training and an external stimulus to the human body. In the process of overcoming this resistance, the body shows its strength and develops its strength quality.

## 4. Conclusions

This paper synthesizes the adaptability of the skeleton to the external environment, and especially introduces the adaptability change of the skeleton to the mechanical stimulus related to sports and its related mechanisms, and modern bone research measurement and evaluation techniques and methods. Restoration by fibrous connective tissue is called fibrous repair. It is also called paralysis scar repair because of the formation of the paralysis scar in the repair. The repairing outcome of a pulled muscle is limited by the degree of muscle injury and the treatment of muscle injury. In exoskeleton design, first, the kinematics principles of the human body are analyzed, and then the joint design of the human skeleton connection mode is simulated. The deflection design conforming to human body structure is adopted to ensure that there is no interference between the human body and the exoskeleton during walking, while improving comfort. As the mechanical load applied to the bone increases, the strain of the bone increases, and when the amount of strain increases to or above a certain limit, the bone can be stimulated to initiate the bone reconstruction process. Thereby, the bone mass is increased and the bone structure is also changed to adapt to the bearing needs, so that the biomechanical properties of the bone are improved and improved. Many sports workers who are engaged in exercise prescriptions to improve bone mass and prevent osteoporosis have a high level of interest and enthusiasm in this regard, which will undoubtedly promote the depth and breadth of research in this area. However, it should be emphasized that we cannot forget the muscles and joints in the basic composition of the human body's motor system while studying bones. In clinical and sports practice, there is an intrinsic and complementary relationship between bone culture and bone health.

## Figures and Tables

**Figure 1:** The initial state of an iterative learning experiment.

**Figure 2:** The initial state of B iterative learning experiments.

**Figure 3:** Iterative learning simulation initial state.

**Figure 4:** Iterative learning simulation output curve.

**Figure 5:** Iterative learning simulation output convergence process.

**Figure 6:** Vertical ground reaction curve.

**Table 1:** Scope of human activity.

	Motion characteristics	Maximum range of motion on foot (°)	Maximum range of motion of joint (°)
Hip joint	Qu	25.56	84
	Stretch	22.15	52
Knee joint	Qu	53.61	32
	Stretch	61.26	56
Ankle joint	Qu	23.51	32
	Stretch	19.52	25

**Table 2:** Calculated results of standing stress on both legs.

Component	Maximum stress (MPa)	Location of maximum stress generation
Back	92.25	Back bracket
Waist	62.21	Dorsal junction
Hip	49.51	Lumbar junction
Thigh	32.12	Deflection point
A lower leg	15.62	Deflection point
Feet	38.16	Ankle joint

**Table 3:** Calculated results of vertical stress of tibia.

Component	Maximum stress (MPa)	Location of maximum stress generation
Back	153.15	Lumbar junction
Lumbar (left)	153.72	Hip junction
Waist (right)	85.62	Hip junction
Hip (left)	92.33	Lumbar junction
Hip (right)	43.51	Lumbar junction
Thigh (left)	106.92	Constraint point
Thigh (right)	125.91	Connection of calf
Crus (left)	26.61	Deflection point
Crus (right)	136.51	Thigh junction
Foot (left)	26.21	Footplate connection
Foot (right)	56.81	Connection of calf

**Table 4:** Calculated parameter value.

Parameter	Value
Population size	*M* = 30
Iteration steps	*K* = 300

## Data Availability

The data used to support the findings of this study are included within the article.
